# A Giant Porencephaly: A Rare Etiology of Pediatric Seizures

This article has been retracted.

**DOI:** 10.7759/cureus.19623

**Published:** 2021-11-16

**Authors:** Rayan A Alzahrani, Ameera F Alghamdi, Mohammed A Alzahrani, Majed A Alghamdi, Malak F Alghamdi, Amjad A Alzahrani, Abdullah M Alghamdi, Manal K Alzahrani, Talal S Alghamdi, Rahaf S Alghamdi, Fahad A Alqarni, Ahmed H Al-Zahrani, Faisal M Al-Hawaj

**Affiliations:** 1 College of Medicine, Al-Baha University, Al-Baha, SAU; 2 College of Medicine, Imam Abdulrahman Bin Faisal University, Dammam, SAU

**Keywords:** epilepsy, case report, mri imaging, porencephaly, seizure

## Abstract

Pediatric convulsive seizure is common and represents a source of major concern and anxiety for the parents. Seizures can have a broad spectrum of etiologies in children, including metabolic, traumatic, developmental, and infectious causes. Depending on the clinical presentation, laboratory testing and neuroimaging may be indicated in the workup of the first unprovoked afebrile seizure. We present a case of a six-year-old boy who was brought to the emergency department by his mother after an episode of convulsion. She reported that he had jerky repetitive movements of all extremities that lasted around two minutes with spontaneous termination. The child did not have a febrile illness. The mother reported no history of similar episodes. Upon examination, the child appeared alert and conscious. No dysmorphic features were evident. Initial laboratory investigations were within the normal limits. The child underwent magnetic resonance imaging for the brain, which demonstrated a large well-defined extra-axial cystic lesion occupying most of the left hemisphere that is connected to the ventricular system. The lesion had no grey-matter lining and it strictly followed the cerebrospinal fluid in all sequences. Such finding represented the diagnosis of a giant left porencephalic cyst. Porencephaly is an extremely rare neurological anomaly that may present with pediatric seizures. Magnetic resonance imaging is the gold standard modality for the diagnosis of porencephaly. The case demonstrated that porencephaly can have a massive size in a patient with normal psychoneurological development.

## Introduction

Pediatric convulsive seizure is common and affects up to 10% of children [1]. It accounts for 1% of all visits to the pediatric emergency [2]. It represents a source of major concern and anxiety for the parents. Seizures can have a broad spectrum of etiologies in children, including metabolic, traumatic, developmental, and infectious causes [3]. While most patients with first-time seizures may not develop further episodes, proper assessment is needed as the seizure may be a manifestation of a serious medical condition or epilepsy. Children presenting with first-time seizures should undergo careful evaluation by experienced clinicians as the diagnostic inaccuracy of seizures is very common [4]. Depending on the clinical presentation, laboratory testing and neuroimaging may be indicated in the workup of the first unprovoked afebrile seizure. Magnetic resonance imaging is the imaging modality of choice in evaluating patients with first-time seizures. It is superior to computed tomography scan to detect structural pathologies [5]. Here, we present a case of a previously well six-year-old boy with a first-time seizure that was found to have a giant porencephalic cyst on imaging.

## Case presentation

We present the case of a six-year-old boy who was brought to the emergency department by his mother after an episode of convulsion. She reported that he had jerky repetitive movements of all extremities that lasted around two minutes with spontaneous termination. He was not responding during the episode. The mother reported that his skin color turned blue. The mother reported that the movement was associated with urinary incontinence and frothy secretions from the mouth. There were no warning signs before the event. The mother reported that the child did not complain of any unpleasant sensation before the spell. The event occurred suddenly while the child was playing with his friend. He was not deprived of sleep before the event. The child appeared tired after the spell and he fell asleep. The child did not have a febrile illness. The mother reported no history of similar episodes.

Regarding the medical history, the child was known to have asthma and eczema. His conditions were well-controlled. There was no history of previous surgeries. The perinatal history was uneventful. He was full-term with a birth weight of 3.8 kg. He was up-to-date with the vaccination schedule. He was not born of a consanguineous marriage. No family history of epilepsy was present. The social history was non-contributory.

Upon examination, the child appeared alert and conscious. No dysmorphic features were evident. He was not pale, jaundiced, or cyanosed. His vital signs included a temperature of 36.5℃, a heart rate of 90 bpm, blood pressure of 80/58 mmHg, and respiratory rate of 23 bpm. His oxygen saturation was 99% on room air. The child had normal speech and comprehension appropriate for his age. His social and behavioral skills were normal. Upper and lower limb examination revealed normal tone and power. His gait was normal. The cardiorespiratory examination was unremarkable. Initial laboratory investigation revealed a hemoglobin of 14.2 g/dL, leukocytes count of 7,000 cells//µL, and platelet count of 390,000/µL. The random blood sugar was within the normal limits. Other biochemical findings, including electrolytes, hepatic, and renal profiles, were within the normal limits (Table 1).

**Table 1:** Summary of the results of laboratory findings.

Laboratory investigation	Unit	Result	Reference range
Hemoglobin	g/dL	14.2	13.0–18.0
White blood cell	1,000/mL	5.3	4.0–11.0
Platelet	1,000/mL	380	140–450
Erythrocyte sedimentation rate	mm/hr	7	0–20
C-reactive protein	mg/dL	0.9	0.3–10.0
Total bilirubin	mg/dL	0.5	0.2–1.2
Albumin	g/dL	3.9	3.4–5.0
Alkaline phosphatase	U/L	48	46–116
Gamma-glutamyltransferase	U/L	19	15–85
Alanine transferase	U/L	17	14–63
Aspartate transferase	U/L	15	15–37
Blood urea nitrogen	mg/dL	9	7–18
Creatinine	mg/dL	0.8	0.7–1.3
Sodium	mEq/L	136	136–145
Potassium	mEq/L	3.7	3.5–5.1
Chloride	mEq/L	104	98–107

Considering the aforementioned findings of unexplained first-time seizure with normal laboratory markers, the child underwent magnetic resonance imaging for the brain to rule out any structural abnormalities. The scan demonstrated a large well-defined extra-axial cystic lesion occupying most of the left hemisphere that is connected to the ventricular system. The lesion had no grey-matter lining and it strictly followed the cerebrospinal fluid in all sequences (Figure 1). Such finding represented the diagnosis of a giant left porencephalic cyst. The patient was referred to the pediatric neurology team. The child was given anticonvulsant therapy (valproic acid) to prevent further seizure episodes. The patient was followed at our institution for six months. He did not develop any further seizures while he was on anticonvulsant therapy.

**Figure 1:** T2-weighted (A and B) and FLAIR (C) MR images of the brain demonstrating a massive left intracranial cyst with CSF density. CSF: cerebrospinal fluid; FLAIR: fluid-attenuated inversion recovery; MR: magnetic resonance.

## Discussion

We presented an interesting case of a child with a first-time seizure due to a giant porencephalic cyst occupying almost all the left hemisphere. Porencephaly is an extremely rare congenital disorder of the brain. Porencephaly can be congenital or acquired after infection, trauma, infarction, or hemorrhage [6]. The size of porencephaly varies significantly from small lesions that may be detected incidentally to significantly large lesions occupying all the cerebral hemispheres [7].

Porencephaly can occur in any lobe. It is typically unilateral in most cases, but cases with bilateral porencephaly have been reported [6]. The clinical manifestation of porencephaly varies and it may be related to the site and size of the lesion. Seizures of different types have been reported in patients with porencephaly. Patients may present with spasticity, psychosis, diplopia, and otorrhea [8-10]. In the present case, the patient had massive porencephaly presenting with a first-time seizure at the age of six years with previously normal neuropsychiatric development.

Magnetic resonance imaging is the gold standard for the diagnosis of porencephaly. As in the present case, it demonstrates an intracranial cystic lesion within the brain that follows the cerebrospinal fluid signal in all sequences and exhibits communication with the ventricular system or the subarachnoid space. The differential diagnoses of porencephaly include schizencephaly, neuroglial cyst, arachnoid cyst, and holoprosencephaly. In contrast to schizencephaly, a porencephalic cyst is not lined by grey matter. Antenatal diagnosis of porencephaly may be possible by third-trimester ultrasound [11]. In the present case, however, the prenatal history was unremarkable.

The surgical management for epilepsy caused by porencephaly can be challenging. It is difficult to choose the optimal surgical approach due to the widespread abnormality that can be detected by electroencephalography. Further, the functional cortical reserve may be limited in such patients. In a case series by Ichikawa et al. [12], they revealed that non-invasive evaluation using single-photon emission computed tomography resulted in determining the origin of the seizure and led to curative surgery with favorable functional outcomes.

## Conclusions

Porencephaly is an extremely rare neurological anomaly. Despite its rarity, clinicians should be aware of this condition and consider it in the differential diagnoses of pediatric seizures. Magnetic resonance imaging is the gold standard modality for the diagnosis of porencephaly. The case demonstrated that porencephaly can have a massive size in a patient with normal psychoneurological development.
